The article "A Novel Chaotic Image Encryption Algorithm Based on Latin Square and Random Shift" was published in 2021. Journal: Comput Intell Neurosci.

# A Novel Chaotic Image Encryption Algorithm Based on Latin Square and Random Shift

**DOI:** 10.1155/2021/2091053

**Published:** 2021-09-06

**Authors:** Xuncai Zhang, Tao Wu, Yanfeng Wang, Liying Jiang, Ying Niu

**Affiliations:** ^1^College of Electrical and Information Engineering, Zhengzhou University of Light Industry, Zhengzhou 450002, China; ^2^College of Architecture Environment Engineering, Zhengzhou University of Light Industry, Zhengzhou 450002, China

## Abstract

To realize the safe transmission of images, a chaotic image encryption algorithm based on Latin square and random shift is proposed. The algorithm consists of four parts: key generation, pixel scrambling, pixel replacement, and bit scrambling. Firstly, the key is generated from the plain image to improve the sensitivity of the encryption method. Secondly, each pixel in each row of the image matrix is moved cyclically to the right, in turn, to change the position of the image pixel and realize pixel position scrambling. Then, a 256-order Latin square matrix composed of a chaotic sequence is used as a lookup table, and the replacement coordinates are calculated based on the image pixel value and the chaotic sequence value, replacing the corresponding coordinate elements in the image matrix. Finally, decompose the bitplane of the image matrix and combine it into two-bit matrices, scramble the two bit matrices, respectively, with the Latin square matrix, recombine the scrambled two-bit matrices, and convert them into decimal to obtain the ciphertext image. In the proposed encryption method, all the Latin square matrices used are generated by chaotic sequences, further enhancing the complexity of the generated Latin square matrix and improving the algorithm's security. Experimental results and security analysis show that the proposed algorithm has good security performance and is suitable for image encryption.

## 1. Introduction

With the rapid development of modern communication technology, more and more digital images are transmitted on social networks. These images carry personal information. Therefore, how to protect this private information has become a research hotspot [1]. Due to the inherent characteristics of strong correlation and high redundancy between adjacent pixels of an image, some traditional encryption methods such as Data Encryption Standard (DES) or Advanced Encryption Standard (AES) are not suitable for performing digital images encryption because traditional encryption algorithms have the disadvantage of low efficiency when encrypting digital images [2].

Because some characteristics of the chaotic system are very suitable for the development of image encryption algorithms, such as sensitivity to initial conditions, unpredictability, and ergodicity, among the currently proposed image encryption methods, chaos systems have been widely used [3–5]. Wang [6] proposed an image encryption method based on a one-dimensional chaotic system, which improved the structure of control parameters and the sensitivity of one-dimensional chaotic mapping and improved its ability to resist differential attacks. Zhou [7] combined two existing one-dimensional chaotic maps and proposed a new one-dimensional chaotic map, which improved the performance against various attacks. However, some inherent shortcomings of one-dimensional chaotic mapping, such as relatively simple structure and small keyspace, are difficult to eliminate. In contrast, high-dimensional chaotic systems have more complex dynamics and high ergodicity, so people apply high-dimensional chaotic systems to image encryption [8–10]. Gan [11] proposed a color image encryption algorithm based on high-dimensional chaos and three-dimensional bit-plane arrangement, which can effectively resist known plaintext attacks and selected plaintext attacks. Zhang [12] proposed a new 3D bit matrix replacement algorithm, and the encryption method developed a new replacement method based on the Chen system to improve the randomness of the scrambling process. However, the encryption scheme is vulnerable to attack by the selected plaintext. Image encryption algorithms based on high-dimensional chaos often scramble the pixels of the image by obtaining the index vector of the chaotic sequence. The security of these scrambling methods only depends on the index vector because the attacker may analyze the difference between the cipher image and the plain image. The relationship to obtain the index vector causes the scrambling operation to be invalid.

In recent years, due to the excellent performance of the Latin square in image encryption methods, it has received extensive attention from researchers. The Latin square is a special square matrix with uniformity. Shannon first pointed out the relationship between the Latin square and cryptography [13]. Latin squares have some good features that are very suitable for image encryption: the number of Latin squares is huge, and the number of Latin squares of the 10^th^ order is about 10^37^, so its keyspace is large and can prevent brute force attacks. The Latin square has a unified histogram, which means that using the Latin square for image encryption can effectively resist statistical analysis. Because of the good characteristics of the Latin square, Wu [14] proposed a symmetric encryption algorithm and designed a new loom-like 2D substitution-permutation network. This network maintains good confusion and diffusion characteristics while also with additional fault tolerance. Panduranga [15] used a chaotic system and Latin square to construct an image encryption method, which was later cracked by Ahmad M. and Ahmad F. [16].

Aiming at the characteristics of chaotic system and Latin square matrix, an image encryption algorithm (LSRS) based on Latin square and random shift is designed. The algorithm is divided into four parts: key generation, pixel scrambling, pixel replacement, and bit scrambling. Latin squares are all produced by chaotic sequences, which further enhances the complexity of Latin squares. In the pixel scrambling part, the cyclic shift step length of the pixel is controlled by the chaotic sequence, which makes the pixel distribution more random. The histogram of the 256-order Latin square matrix is evenly distributed; using it as a lookup table to replace the pixels can effectively increase the Shannon entropy of the cipher image. At the same time, the image pixel value and the rounded chaotic sequence jointly calculate the coordinates of the replaced pixels, which effectively improves the randomness of the algorithm, through the Latin square matrix to scramble the bit plane of the image matrix to enhance the security of the algorithm. The security analysis of the encrypted cipher image shows that the LSRS algorithm has good security performance and is suitable for practical applications.

The rest of this article is organized as follows: in Section 2, the related concepts of Latin squares and chaotic systems are introduced.  Section 3 gives the detailed scheme of the LSRS method.  Section 4 analyzes the safety of the proposed method. Finally, the conclusions are given in Section 5.

## 2. Related Work

### 2.1. Latin Square

The famous mathematician and physicist Euler used the Latin alphabet as the symbol of the elements in the Latin square, and the Latin square got its name. For an *N* × *N* matrix with only *N* different elements and each element appears only once in any row or column, the matrix is called a Latin square matrix. The application of the Latin square matrix is to double control the row vector and column vector of the image matrix to promote the uniform distribution of pixels and improve the balance of pixels in the matrix.  Figure 1 shows examples of Latin squares with different symbol sets.

### 2.2. Hyperchaotic Lorenz System

The hyperchaotic Lorenz system has multiple positive Lyapunov exponents, has a high keyspace, and can improve the confidentiality performance of the encryption algorithm [17]. The dynamic formula of hyperchaotic Lorenz is

(1) $$\begin{array}{c} \left\{\begin{array}{c} \dot{x}=-a\left(y-x\right)+w,\\ \dot{y}=cx-y-xz,\\ \dot{z}=xy-bz,\\ \dot{w}=-yz+rw, \end{array}\right. \end{array}$$

where *a*, *b*, *c,* and *r* are all control parameters, and when *a* = 10, *b* = 8/3, *c* = 28, and −1.52 ≤ *r* ≤ −0.06, formula (1) is in a hyperchaotic state. When *r* = −1, the four Lyapunov exponents in formula (1) are, respectively, *λ*_1_ = 0.3381, *λ*_2_ = 0.1586, *λ*_3_ = 0, *λ*_4_ = −15.1752, as shown in Figure 2 for the phase of the hyperchaotic Lorenz in the hyperchaotic state.

## 3. Encryption Scheme

In the encryption algorithm, **P** represents a plain image with a size of *N* × *N*, and ***C*** represents the corresponding cipher image. The frame diagram of the encryption scheme is shown in Figure 3.

### 3.1. Generate Key

The plain image to generate the key can associate the plain image with the cipher image and enhance the sensitivity of the key. The method of generating the key in this paper is as follows: divide the input image matrix **P** into four blocks; calculate the sum of the elements in each matrix; and obtain *LL*_1_, *LL*_2_, *LL*_3_, and *LL*_4_ to generate keys *x*_0_, *y*_0_, *z*_0_, and *w*_0_. The method of its generation is

(2) $$\begin{array}{c} \left\{\begin{array}{c} LL1=\mathrm{mod}\left(\overset{\text{floor}\left(N/2\right)}{\underset{i=1}{\sum }}\overset{\text{floor}\left(N/2\right)}{\underset{j=1}{\sum }}P\left(i,\;j\right),256\right),\\ LL2=\mathrm{mod}\left(\overset{\text{floor}\left(N/2\right)}{\underset{i=1}{\sum }}\overset{N}{\underset{j=\text{floor}\left(N/2\right)+1}{\sum }}P\left(i,\;j\right),256\right),\\ LL3=\mathrm{mod}\left(\overset{N}{\underset{i=\text{floor}\left(N/2\right)+1}{\sum }}\overset{\text{floor}\left(N/2\right)}{\underset{j=1}{\sum }}P\left(i,\;j\right),256\right),\\ LL4=\mathrm{mod}\left(\overset{N}{\underset{i=\text{floor}\left(N/2\right)+1}{\sum }}\overset{N}{\underset{j=\text{floor}\left(N/2\right)+1}{\sum }}P\left(i,\;j\right),256\right), \end{array}\right. \end{array}$$

where *LL* = mod (*x*, *y*) returns the remainder after dividing *x* by *y*, *x* is the dividend, *y* is the divisor, and floor (*x*) means rounding the elements of *x* to the negative infinity. The key generation method is

(3) $$\begin{array}{c} \left\{\begin{array}{c} x_{0}=\frac{\left|\left(LL1-\text{bitxor}\left(LL2,\text{bitxor}\left(LL3,LL4\right)\right.\right)\right|}{256},\\ y_{0}=\frac{\left|\left(LL2-\text{bitxor}\left(LL1,\text{bitxor}\left(LL3,LL4\right)\right.\right)\right|}{256},\\ z_{0}=\frac{\left|\left(LL3-\text{bitxor}\left(LL1,\text{bitxor}\left(LL2,LL4\right)\right.\right)\right|}{256},\\ w_{0}=\frac{\left|\left(LL4-\text{bitxor}\left(LL1,\text{bitxor}\left(LL2,LL3\right)\right.\right)\right|}{256}, \end{array}\right. \end{array}$$

where bitxor represents the bitwise exclusive or between two values and |*x*| represents rounding of *x*. Input the generated keys *x*_0_, *y*_0_, *z*_0_, and *w*_0_ into the chaotic system, and iterate 3*M* × *M* times (when *N* < 256, *M* = 256; when *N* ≥ 256, *M* = *N*); the chaotic sequence *X*, *Y*, *Z*, and *W* used for pixel scrambling, pixel replacement, and bit scrambling is obtained.

### 3.2. The Generation of Latin Square Matrix

Given two sequences **Q**_1_ and **Q**_2_ of equal length and sorting them respectively, the corresponding index sequences **Q**_**seed**_ and **Q**_**shift**_ are obtained. According to Algorithm 1 [18], generate Latin square matrix ***L***.

### 3.3. Pixel Scrambling

Pixel scrambling can effectively break the correlation between adjacent pixels and improve the security of encryption algorithms. In this paper, adaptive shifting is used to realize pixel position scrambling, and each pixel in each row (column) is cyclically moved to the right in order from left to right. The step length of each pixel shift in the same row (column) is controlled by the element value of the chaotic sequence, and it is also affected by the previous pixels. This method can increase the complexity of scrambling; even if a chaotic sequence of a certain length is deciphered, it is difficult to restore the image pixels after scrambling correctly. The *N* *×* *N* elements before the chaotic sequence **X** and **Y** are, respectively, intercepted, and two equal sequences **Q**_**r1**_ and **Q**_**r2**_ are obtained. The preprocessing is performed according to formula (4) to get the sequences **Q**_**u1**_ and **Q**_**u2**_, and they are, respectively, converted into *N* × *N.* The matrix **Q**_**row**_ and the matrix **Q**_**col**_ are used for row scrambling and column scrambling of the input image matrix:

(4) $$\begin{array}{c} \left\{\begin{array}{c} Q_{u1}\left(k\right)=\mathrm{mod}\left(Q_{r1}\left(k\right)\times 2^{32},N\right),\\ Q_{u2}\left(k\right)=\mathrm{mod}\left(Q_{r2}\left(k\right)\times 2^{32},\;N\right), \end{array}\right. \end{array}$$

where *k* = 1, 2, 3, ..., *N*.

First, use the matrix **Q**_row_ to scramble each row of the image matrix **P** to obtain the matrix **P**′ , and then use the matrix **Q**_col_ to scramble each column of the matrix **P**′ to get the scrambled matrix **P**_*s*_.  Figure 4 shows an example of the scrambling process of the image matrix **P**. To better explain this scrambling method, the first row of the image matrix **P** and the first row of the matrix Qrow shown in Figure 4 are taken as an example to introduce the adaptive scrambling process in detail, where the adaptive shifting process of the remaining rows (columns) of the image matrix **P** is similar to the scrambling process of the first row of adaptive shifting and will not be described in detail. The scrambling method is as follows:

1. The sequence of the first row of the image matrix **P** is sequence **T** = [101, 33, 44, 55, 12], and the sequence of the first row of the matrix **Q**_row_ used to shift the pixels is sequence **U** = [2, 0, 4, 2, 3];
2. The first element in the sequence **T** is 101, and its first element in the corresponding pixel shift sequence **U** is 2; then, the first element 101 in the sequence **T** is cyclically moved two positions to the right, getting sequence **T**_1_ = [33, 44, 101, 55, 12];
3. The second element in sequence **T**_1_ is 44, and its second element in the corresponding pixel shift sequence **U** is 0; then, the second element 44 in sequence **T**_1_ is cyclically moved zeros positions to the right, getting sequence **T**_2_ = [ 33, 44, 101, 55, 12];
4. The third element in sequence **T**_2_ is 101, and its third element in the corresponding pixel shift sequence **U** is 4; then, the third element 101 in sequence **T**_2_ is cyclically moved four positions to the right, getting sequence **T**_3_ = [ 33, 101, 44, 55, 12];
5. The fourth element in sequence **T**_3_ is 55, and its fourth element in the corresponding pixel shift sequence **U** is 2; then, the fourth element 55 in sequence **T**_3_ is cyclically moved two positions to the right, getting sequence **T**_4_ = [55, 33, 101, 44, 12];
6. The fifth element in sequence **T**_4_ is 12, and its fifth element in the corresponding pixel shift sequence **U** is 3; then, the fifth element 12 in sequence **T**_4_ is cyclically moved three positions to the right, getting sequence **T**_5_ = [55, 33, 12, 101, 44];
7. Repeat the scrambling processes (1)–(6) to the remaining rows of the image matrix **P**, until each row is scrambled to obtain the matrix **P**′.
8. Similar to processes (1)–(7), use matrix **Q**_**col**_ to scramble each column of matrix **P**′ to obtain the scrambled matrix **P**_**S**_.

### 3.4. Pixel Replacement

In the encryption algorithm, replacing the pixels of the plain image can effectively hide the original information of the plain image. However, some encryption algorithms use the replacement method of addition, subtraction, and xor, which is too simple to protect the image information effectively. To solve this defect, generate a 256-order Latin square matrix, and use the elements in this Latin square matrix to replace the pixels of the image. The number of Latin squares of order 256 is about 256! ≈ 2^1684^, so its keyspace is large enough, and its histogram is evenly distributed, which is difficult to crack using statistical attack analysis.

Given two sequences **Q**_*t1*_ and **Q**_*t2*_ of length 256, generate a Latin square matrix **L**_table_ as a lookup table. According to formula (5), get **Q**_**s**1_ and **Q**_**s**2_ and respectively converted into *N* × *N* matrices **L**_*c*_ and **L**_*r*_:

(5) $$\begin{array}{c} \left\{\begin{array}{c} Q_{s1}=\mathrm{mod}\left(Z\left.\left[513\;:\left(512+N\times N\right)\right)\right]\times 2^{32},\;256\right),\\ Q_{s2}=\mathrm{mod}\left(Z\left[\left(513+N\times N\right):\left(512+2\times N\times N\right)\right]\times 2^{32},\;256\right), \end{array}\right. \end{array}$$

where **Z**[*a*: *b*] means to intercept the elements whose index values are between *a* and *b* from the sequence **Z** (including the elements corresponding to the index values *a* and *b*). Through the matrix **L**_*c*_ and the corresponding coordinate element of the image matrix to be replaced to do the addition operation, take the remainder so that the elements in the resulting remainder matrix **L**_*c*_′ are between 0 and 255. Using **L**_*c*_′ as the row coordinate index matrix and the matrix **L**_**r**_ as the column coordinate index matrix, from the lookup table, search the corresponding element for replacement, and get the pixel replacement matrix **P**_*r*_. The replacement method is **P**_*r*_ (*i*, *j*) = **L**_**table**_ (**L**_*c*_′ (*i*, *j*), **L**_*r*_ (*i*, *j*)), where **L**_*c*_′ (*i*, *j*) indicates the row index and **L**_*r*_ (*i*, *j*) indicates the column index.  Algorithm 2 is the Latin square replacement process.

### 3.5. Bit Scrambling

The pixel value of grayscale images ranges from 0 to 255, and an 8-bit binary sequence can represent each pixel. Therefore, the grayscale image can be decomposed into eight bit-planes, where the *i*th bit plane is composed of the *i*th bit of all pixels (*i* = 1, 2, ..., 8). The high bit-plane contains the visual information of the plain image, and the low-bit plane contains the detailed information of the plain image [19]. Mixing the bits in the high-bit plane and the low-bit plane of the plain image can hide the information of the plain image and improve the security of the algorithm.

To better scramble the bits of the image, we decompose the image into eight bit-planes and then recombine and scramble them. First, the image matrix **P** is decomposed into eight bit-planes **P** (1)–**P** (8). Secondly, the four bit-planes **P** (1), **P** (3), **P** (5), and **P** (7) of the image matrix **P** combine into a 2*N* × 2*N* bit matrix **PA**, and the four bit-planes **P** (2), **P** (4), **P** (6), and **P** (8) of the image matrix **P** are combined into a 2*N* × 2*N* bit matrix **PB**. Then, intercept 8*N* elements from the chaotic sequence **W** and divide them into four equal sequences **QD**_1_, **QD**_2_, **QD**_3_, and **QD**_4_. Finally, use the sequences **QD**_1_ and **QD**_2_ to generate the Latin square matrix **LH**_1_, and use the sequences **QD**_3_ and **QD**_4_ to generate the Latin square matrix **LH**_2_, **LH**_1_, and **LH**_2_, respectively used for bit scrambling of matrix **PA** and matrix **PB**.  Figure 5 shows the bit plane of the image matrix **P** is scrambled. Decompose the image matrix P into eight bit-planes, and the bit plane **P** (1) as shown in Figure 5(a). Arrange according to the method shown in Figure 5(b) to obtain a bit matrix **PA** and a bit matrix **PB**. Use the matrix **LH**_1_ to perform row scrambling on the bit matrix **PA** to get **PA**′ , use **LH**_2_ to perform column scrambling on the bit matrix **PB** to obtain **PB**′ , as shown in Algorithm 3, the scrambling process. The bit matrix **PA**′ and bit matrix **PB**′ as shown in Figure 5(c) are obtained. Finally, through the bit matrix **PA**′ and bit matrix **PB**′ recombined into eight bit-planes and converted to decimal, the resulting image matrix **P**_**d**_ is shown in Figure 5(d).

### 3.6. Image Encryption Process

The LSRS algorithm proposed in this paper consists of four parts: key generation, pixel scrambling, pixel replacement, and bit scrambling. The steps of the encryption algorithm are described as follows:

**Step 1 .**

Through the image matrix **P** of size *N* × *N*, generate the initial parameters *x*_0_, *y*_0_, *z*_0_, and *w*_0_ of the *keys*. Input the generated *keys* parameters *x*_0_, *y*_0_, *z*_0_, and *w*_0_ into the hyperchaotic Lorenz system, iterate 999 + 3*M* × *M* times (when *N* *<* 256, *M* *=* 256, when *N* *≥* 256, *M* *=* *N*), and discard the first 999 times; the chaotic sequence **X**, **Y**, **Z**, **W** was obtained.

**Step 2 .**

Intercept the first *N* × *N* elements of the chaotic sequence **X** and **Y**, respectively, as the sequences **Q**_*r1*_ and **Q**_*r2*_; preprocess them according to formula (4); convert them, respectively, into *N* × *N* matrix **Q**_row_ and matrix **Q**_col_; and perform row scrambling and column scrambling of matrix **P** on the image to obtain the scrambling image matrix **P**_*s*_.

**Step 3 .**

Intercept the first 512 elements of the chaotic sequence **Z**, divide them into two equal sequences **Q**_*t1*_ and **Q**_*t2*_, and use them to generate a Latin square matrix **Q**_table_ as a lookup table. According to formula (5) to obtain **Q**_*s1*_ and **Q**_*s2*_, respectively convert into *N* × *N* matrices **L**_*c*_ and **L**_*r*_. Through the matrix **L**_*c*_ and the corresponding coordinate element of the image matrix to be replaced to do the addition operation, take the remainder so that the elements in the resulting remainder matrix **L**_*c*_^**'**^ are between 0 and 255. The matrix **L**_*c*_^**'**^ and the matrix **L**_*r*_ form a two-dimensional index matrix, and the index matrix is used to select elements from the corresponding coordinates in the matrix **Q**_table_ and replace the elements in the matrix **P**_*s*_ to obtain the pixel replacement matrix **P**_*r*_.

**Step 4 .**

Intercept 8*N* elements from the chaotic sequence **W** , divide them into four sequences **QD**_1_, **QD**_2_, **QD**_3_, and **QD**_4_ of equal length. Use **QD**_1_ and **QD**_2_ to generate Latin square matrix **LH**_1_, **QD**_3_, and **QD**_4_ to generate Latin square matrix **LH**_2_. Divide the matrix **P**_r_ into eight bit-planes **P** (1)–**P** (8), where the four bit-planes **P** (1), **P** (3), **P** (5), and **P** (7) are combined into a 2*N* *×* 2*N* bit matrix **PA**, and **P** (2), **P** (4), **P** (6), and **P** (8) four bit-planes are combined into a 2*N* *×* 2*N* bit matrix **PB**. Through matrix **LH**_1_ to scramble the rows of matrix **PA**, **LH**_2_ performs column scrambling on the matrix **PB**. The scrambled matrix **PA**′ and matrix **PB**′ are, respectively, divided into four bit-planes, and the resulting bit planes are combined into a bit plane matrix *P*_bit_′. Convert the elements in the bit plane matrix *P*_bit_′ to decimal data and finally obtained the cipher image **C**.

The reverse process of the encryption algorithm is the decryption process, which will not be repeated.

### 3.7. Simulation Results

In order to study the confidentiality performance of the LSDR method, use MATLAB 2019a to simulate the encryption algorithm. The configuration environment of the computer is Windows 10, 8.00 GB RAM, Intel (R) Core (TM) i7-4510 CPU @ 2.00 GHz.  Figure 6 shows the plain image, cipher image, and decrypted image of Lena, Boat, Hill, and Peppers. By directly observing the cipher image, no valid information can be identified, so the algorithm is feasible.

## 4. Experimental Results and Performance Analysis

### 4.1. Keyspace

The key is the most critical part of the encryption scheme. The larger the keyspace, the stronger the ability to resist brute force attacks, so the key should have enough space to resist brute force attacks. In theory, when the keyspace reaches 2^100^, it is enough to resist the brute force attacks that currently exist. The algorithm proposed has four parameters *x*_0_, *y*_0_, *z*_0_, and *w*_0_. The calculation accuracy of these four parameters is 10^−15^, and the keyspace can reach 10^60^ ≈ 2^190^, which is much larger than 2^100^. Therefore, the keyspace of the LSRS algorithm is large enough to protect the security of the image.

### 4.2. Differential Attack Analysis

Differential attack refers to studying the influence of the difference between plain images on their cipher image and establishing a relationship between the plain image and its corresponding cipher image, thereby cracking the encryption method. The number of Pixel Change Rate (NPCR) and Unified Pixel Average Change Intensity (UACI) are two methods to test whether the encryption method can resist differential attacks [23]. NPCR reflects the ratio of the number of unequal pixels in the same position of two images to the number of all pixels in the image. UACI is the overall average change density, which represents the average change intensity of the planar image. The ideal values of NPCR and UACI are, respectively, 99.6094% and 33.4635%. Assuming that **P**_1_ and **P**_2_ are two cipher images and their plain images only have a one-bit difference, their NPCR and UACI values are calculated as shown in the following formula:

(6) $$\begin{array}{c} \left\{\begin{array}{c} \text{NPCR}=\frac{\sum_{i=1}^{M}\sum_{j=1}^{N}D_{\left(i,j\right)}}{M\times N}\times 100\%,\\ \text{UACI}=\frac{\sum_{i=1}^{M}\sum_{j=1}^{N}\left|P_{1}\left(i,j\right)-P_{2}\left(i,j\right)\right|}{255\times M\times N}\times 100\%, \end{array}\right. \end{array}$$

where **P**_1_ (*i*, *j*) ≠ **P**_2_ (*i*, *j*), *D* (*i*, *j*) = 1; otherwise, *D* (*i*, *j*) = 1.

Taking Lena image as an example, Table 1 compares the test results of NPCR and UACI under different algorithms. It can be seen that the encryption method we propose can resist differential attacks more effectively.

### 4.3. Key Sensitivity Analysis

To ensure the security of the encryption algorithm, the encryption algorithm should be highly sensitive to the input key. When the wrong key is entered to decrypt the cipher image, the output is an image that cannot identify any information. The LSDR algorithm proposed in this paper uses the Lena image as a test. First, input the image into the LSDR algorithm to obtain the keys = [*x*_0_, *y*_0_, *z*_0_, *w*_0_] and the cipher image. The element *x*_0_ in the keys is slightly modified by adding 1 to the 15^th^ digit after the decimal point and then using the modified keys′  = [*x*_0_ + 10^−15^, *y*_0_, *z*_0_, *w*_0_] to decrypt.  Figure 7 shows the decrypted image under the correct key and the decrypted image obtained after modifying the key parameters *x*_0_, *y*_0_, *z*_0_, and *w*_0_, respectively. It can be seen that even if the decryption key changes slightly, the correct decrypted image cannot be obtained. Therefore, the key sensitivity in the LSDR algorithm is high enough to resist all types of brute force attacks.

### 4.4. Histogram Analysis

The histogram can intuitively reveal the distribution of pixel values in the image. Cipher image has a unified histogram, which can effectively resist statistical analysis, making it difficult for an attacker to obtain valuable information. The more even the pixel distribution in the cipher image, the more ideal the encryption algorithm. As shown in Figure 8, the plain image is input to the LSRS algorithm for encryption, and the histogram of the cipher image obtained is evenly distributed. In addition, the flatness of the histogram can be quantified numerically. The standard method is the chi-square test [24], which is defined as

(7) $$\begin{array}{c} X^{2}=\sum_{0}^{255}\frac{{\left(V_{i}-V_{0}\right)}^{2}}{V_{0}}, \end{array}$$

where *V*_0_=((*M* × *N*)/256), *M* × *N* is the size of the image, and *V*_*i*_ and *V*_o_, respectively, represent the actual and expected frequency of each gray level. Set the significance level as *α* = 0.05. If *X*_test_^2^ is less than *X*_*α*_^2^  = 293.25 [25], the histogram can be considered to be uniformly distributed. In this paper, test the three images of Lena, Boat, and Hill. From the results in Table 2, it can be seen that the proposed method is lower than the theoretical value of 293.25. Therefore, it can be considered that the program passed the chi-square test.

### 4.5. Correlation Analysis

The adjacent pixels of the plain image have a high correlation in the horizontal, vertical, and diagonal directions. The ideal encryption algorithm can reduce the correlation of adjacent pixels in the cipher image, thereby effectively resisting statistical attacks. The correlation coefficient calculation formula is

(8) $$\begin{array}{c} \left\{\begin{array}{c} E\left(x\right)=\frac{1}{N}\sum_{i=1}^{N}x_{i},\\ D\left(x\right)=\frac{1}{N}\sum_{i=1}^{N}{\left(x_{i}-E\left(x\right)\right)}^{2},\\ \mathrm{cov}\left(x,y\right)=\frac{1}{N}\sum_{i=1}^{N}\left(\left(x_{i}-E\left(x\right)\right)\left(y_{i}-E\left(y\right)\right)\right),\\ \rho_{xy}=\frac{\mathrm{cov}\left(x,y\right)}{\sqrt{D_{x}}\times \sqrt{D_{y}}}, \end{array}\right. \end{array}$$

where *x* and *y* are pixel values, cov (*x*, *y*) is the covariance, *D* (*x*) is the variance, *E* (*x*) is the mean, and *ρ*_*xy*_ is the correlation coefficient.

To analyze the correlation between adjacent pixels in the plain image and the cipher image, take Lena image as an example, randomly select 2000 pairs of adjacent pixels in the plain image and the cipher image to test. As shown in Table 3, the distribution of adjacent pixels in the plain image of Lena is highly concentrated, so the correlation between adjacent pixels of the plain image is very high. The distribution of adjacent pixels in the cipher image of Lena is random, which means that after encryption, the correlation between adjacent pixels of the cipher image of Lena is low. By comparing with the other three encryption methods, the results of the LSDR algorithm are also satisfactory.

### 4.6. Global Shannon Entropy and Local Shannon Entropy

Global Shannon Entropy (GSE) is a disordered statistical measure that reflects the randomness of information. The calculation formula of GSE [26] is

(9) $$\begin{array}{c} H\left(m\right)=-\sum_{i=0}^{Q}P\left(m_{i}\right)\log_{2}\;P\left(m_{i}\right), \end{array}$$

where *Q* is the gray level of the image. For 8-bit grayscale images, *Q* = 255. *m*_*i*_ is the *i*th gray value on the image, and *P*(*m*_*i*_) is the probability of *m*_*i*_. In an entirely randomly generated image, the ideal value of GSE is 8. The closer the GSE of the image is to 8, the more random the image information.

Local Shannon Entropy (LSE) is proposed by Wu [27] to measure the randomness of encrypted images. For image **P**, randomly select *k* nonoverlapping image blocks *S*_1_, *S*_2_,…, *S*_*k*_ and *T*_*B*_ pixels, and LSE is defined as

(10) $$\begin{array}{c} \bar{H_{k,\;T_{B}}}\left(P\right)=\sum_{i=1}^{k}\frac{H\left(S_{i}\right)}{k}, \end{array}$$

where *H* (*S*_*i*_) is the Shannon entropy of the image block *S*_*i*_. This article selects (*k*, *T*_*B*_) = (30, 1936) to test the cipher image. If the value of LSE is in the interval [*h*_left_^*l∗α*^, *h*_right_^*l∗α*^], it means that the randomness is passed inspection; it can be considered that the cipher image has high randomness. Tested by encrypting the images in the USC-S IPI image database, the test results are shown in Table 4. It can be seen from Table 4 that after LSRS algorithm encryption, the GSE of the cipher image is very close to the ideal value, and most of the cipher images have passed the LSE critical value test. It can be considered that the generated cipher images have high randomness.

### 4.7. Antinoise Attack Analysis and Cropping Attack Analysis

Digital images may lose data or be disturbed by noise due to various reasons during the transmission process. An effective image encryption method can reconstruct an identifiable decrypted image in the case of noise interference or data loss. Add 1%, 5%, and 10% salt and pepper noise to cipher image of Lena, and then decrypt it. As shown in Figure 9, even if a certain salt and pepper noise is added to the cipher image, the information of the decrypted image can still be identified. As shown in Figure 10, cipher images of Lena images are cropped 1/64, 1/16, and 1/4, respectively, and then decrypted, which can identify the information of the decrypted image, so the algorithm can resist the analysis of cropping attacks.

### 4.8. Efficiency Analysis

The efficiency of image encryption is also one of the important indicators to measure the quality of image encryption methods. The main time-consuming parts of the LSRS algorithm are the iteration of the chaotic sequence, Latin square scrambling, Latin square replacement, and Latin square diffusion. In the simulation, take Lena as an example, we compared the encryption time of four different algorithms.  Table 5 lists the running time of each algorithm, and the simulation result shows that the encryption efficiency of the LSRS algorithm is higher.

## 5. Conclusion

This paper proposes a novel chaotic image encryption algorithm based on Latin square and random shift. The LSRS algorithm adopts the structure of pixel scrambling-replacement-bit scrambling. The generation of Latin squares in the encryption process is related to the chaotic sequence, which improves the security of the entire encryption system. Since the histogram of the Latin square is evenly distributed, use the elements in the Latin square lookup table to replace pixels, and the algorithm can effectively resist differential attacks. Each cipher image corresponds to a Latin square lookup table, which increases the difficulty of the algorithm to decipher. The simulation results prove the safety and effectiveness of the LSRS algorithm.

## Figures and Tables

**Figure 1:** Latin square example. (a) 3 × 3. (b) 4 × 4. (c) 5 × 5. (d) 9 × 9.

**Figure 2:** Phase diagram of the hyperchaotic Lorenz system. (a) *x*_*n*_*-y*_*n*_ phase diagram, (b) *y*_*n*_*-w*_*n*_ phase diagram, (c) *x*_*n*_*-z*_*n*_ phase diagram, (d) *y*_*n*_*-z*_*n*_ phase diagram, (e) *x*_*n*_*-w*_*n*_ phase diagram, and (f) *z*_*n*_*-w*_*n*_ phase diagram.

**Figure 3:** Block diagram of the encryption scheme.

**Figure 4:** Example of scrambling of image matrix (*P*).

**Figure 5:** The bit plane of the image matrix (P) is scrambled. (a) Decompose the bit plane of the image matrix (P) to obtain the bit plane matrix **P**_bit_, (b) the bit matrix *PA* and the bit matrix *PB*, (c) the bit matrix *PA*′ and the bit matrix *PB*′, and (d) the bit plane matrix *P*_bit_′ and image matrix *P*_*d*_.

**Figure 6:** Plain image, cipher image, and decrypted image. (a) Plain image of Lena. (b) Cipher image of Lena. (c) Decrypted image of Lena. (d) Plain image of Boat. (e) Cipher image of Boat. (f) Decrypted image of Boat. (g) Plain image of Hill. (h) Cipher image of Hill. (i) Decrypted image of Hill.

**Figure 7:** Plain image of Lena and the decrypted image after different parameters of the decryption key are changed: (a) plain image of Lena, (b) correct keys, (c) *x*_0_ + 10^−15^, (d) *y*_0_ + 10^−15^, (e) *z*_0_ + 10^−15^, and (f) *w*_0_ + 10^−15^.

**Figure 8:** The histogram of the plain image and the corresponding cipher image. (a) The histogram of the Lena plain image. (b) The histogram of the Boat plain image. (c) The histogram of the Hill plain image. (d) The histogram of the Lena cipher image. (e) The histogram of the Boat cipher image. (f) The histogram of the Hill cipher image.

**Figure 9:** The encrypted image and the decrypted image after salt and pepper noise attack. (a) 1% attack encrypted image, (b) 5% attack encrypted image, (c) 10% attack encrypted image, (d) 1% attack decrypted image, (e) 5% attack decrypted image, and (f) 10% attack decrypted image.

**Figure 10:** The cropped encrypted image and decrypted image. (a) The 1/64 cropping encrypted image, (b) the 1/16 cropping encrypted the image, (c) the 1/4 cropping the encrypted image, (d) the 1/64 cropping decrypted image, (e) the 1/16 cropping decrypted image, and (f) the 1/4 cropping decrypted image.

**Algorithm 1:** Latin square produces **L** = Latin (**Q**_1_, **Q**_2_).

**Algorithm 2:** Latin square substitution **P**_*r*_ = Replace (**P**, **L**_*c*_′ (*i*, *j*), **L**_*r*_, **L**_table_).

**Algorithm 3:** Bit scrambling **P**_**d**_ = diffusion (**P**, **LH**_1_, **LH**_2_).

**Table 1:** The Lena image test results in different schemes.

Index (%)	Ideal value	Ours	[20]	[21]	[22]
NPCR	99.6094	99.6101	99.65	99.61	99.66
UACI	33.4635	33.4583	33.56	33.48	33.49

**Table 2:** **x**^2^ test results.

Image	Lena	Boat	Hill	Peppers
*x*_0.05_^2^	293.25	293.25	293.25	293.25
*x*_test_^2^	257.3516	237.9063	222.5469	270.8047
Decision	Pass	Pass	Pass	Pass

**Table 3:** Correlation analysis.

	Horizontal (%)	Vertical (%)	Diagonal (%)
Plain image Lena	0.9618	0.9854	0.9618
Our method	0.0023	0.0158	0.0147
Ref. [20]	−0.0226	0.0041	0.0368
Ref. [21]	−0.0059	−0.0146	0.0211
Ref. [22]	0.0220	0.01792	7*E*−06

**Table 4:** GSE and LSE test analysis.

Image	GSE	LSE	LSE critical value *k* = 30, *T*_*B*_^*Q*=256^*∗*^^ = 1936		
			*h*_left_^*l∗*0.001^=7.9015	*h*_left_^*l∗*0.01^=7.9017	*h*_left_^*l∗*0.05^=7.9019
			*h*_right_^*l∗*0.001^=7.9034	*h*_right_^*l∗*0.01^=7.9032	*h*_right_^*l∗*0.05^=7.9030
			0.001-level	0.01-level	0.05-level
5.1.09	7.9976	7.9027	Pass	Pass	Pass
5.1.10	7.9973	7.9022	Pass	Pass	Pass
5.1.11	7.9976	7.9030	Pass	Pass	Pass
5.1.12	7.9975	7.9033	Pass	Pass	Pass
5.1.13	7.9972	7.9021	Pass	Pass	Pass
5.1.14	7.9970	7.9024	Pass	Pass	Pass
5.2.08	7.9992	7.9034	Pass	No	No
5.2.09	7.9994	7.9035	No	No	No
5.2.10	7.9992	7.9028	Pass	Pass	Pass
7.1.01	7.9993	7.9032	Pass	Pass	No
7.1.02	7.9994	7.9019	Pass	Pass	Pass
7.1.03	7.9993	7.9036	No	No	No
7.1.04	7.9993	7.9020	Pass	Pass	Pass
7.1.05	7.9992	7.9054	No	No	No
7.1.06	7.9993	7.9020	Pass	Pass	Pass
7.1.07	7.9993	7.9025	Pass	Pass	Pass
7.1.08	7.9994	7.9028	Pass	Pass	Pass
7.1.09	7.9993	7.9049	No	No	No
7.1.10	7.9993	7.9030	Pass	Pass	Pass
7.2.01	7.9998	7.9020	Pass	Pass	Pass

**Table 5:** Running time of four different algorithms.

Algorithm	Ours	[20]	[21]	[22]
Time (second)	0.325	0.613	0.3243	0.425

## Data Availability

The data used to support the findings of this study are included within the article.
